The article "Online Anomaly Detection of Industrial IoT Based on Hybrid Machine Learning Architecture" was retracted in 2023. Reasons: signs of a paper mill; suspected computer-generated content; unreliable results or conclusions; concerns about the data.

# Online Anomaly Detection of Industrial IoT Based on Hybrid Machine Learning Architecture

**DOI:** 10.1155/2022/8568917

**Published:** 2022-04-30

**Authors:** Jia Guo, Yue Shen

**Affiliations:** ^1^Zhengzhou Sias University, Department of Electronics and Information, Zhengzhou 451100, China; ^2^Henan Geology Mineral College, Zhengzhou 451464, China

## Abstract

Industrial IoT (IIoT) in Industry 4.0 integrates everything at the level of information technology with the level of technology of operation and aims to improve Business to Business (B2B) services (from production to public services). It includes Machine to Machine (M2M) interaction either for process control (e.g., factory processes, fleet tracking) or as part of self-organizing cyber-physical distributed control systems without human intervention. A critical factor in completing the abovementioned actions is the development of intelligent software systems in the context of automatic control of the business environment, with the ability to analyze in real-time the existing equipment through the available interfaces (hardware-in-the-loop). In this spirit, this paper presents an advanced intelligent approach to real-time monitoring of the operation of industrial equipment. A hybrid novel methodology that combines memory neural networks is used, and Bayesian methods that examine a variety of characteristic quantities of vibration signals that are exported in the field of time, with the aim of real-time detection of abnormalities in active IIoT equipment are also used.

## 1. Introduction

The industry sector within Industry 4.0 introduces and uses the Internet of Things in all its functions, which has contributed to the implementation of severe innovative leaps [1, 2]. Each part of the industrial ecosystem that participates in the production process is accompanied by a massive volume of generated data, which describe its regular operation while also containing frequent anomalies related to every day or improper use [3]. The ability to detect abnormalities in the equipment process in real-time has a significant impact on the overall operation of the industrial environment while offering stability and reliability during its management. [4].

This possibility, especially when attempted without human supervision, is complex as it depends on many factors. Initially, the key to this process is to determine the exact boundary between normal and abnormal operations, which presents the most significant difficulty in this analysis [5]. To select the appropriate anomaly detection technique, several factors must be weighed. The most important is the nature of the data produced, i e., binary, continuous in time, or discrete values and their relationship. The availability of data and the determination of the type of deviant behavior should also be specified. More specifically, it should be determined whether it refers to an anomaly of a point pattern or whether the specific behavior is under conditions [6].

The article "Online Anomaly Detection of Industrial IoT Based on Hybrid Machine Learning Architecture" was retracted in 2023. Reasons: signs of a paper mill; suspected computer-generated content; unreliable results or conclusions; concerns about the data.

Point anomaly refers to detecting a point whose value differs from the rest of the data set. The type of data set to which this anomaly refers is the one where its values have a specific range and, in regular operation, do not exceed the maximum and minimum value that it determines. Therefore, a sharp increase or decrease in a value that simultaneously exceeds these limits can be described as an abnormal behavior of the equipment or operation. Such anomalies are best detected before processing the data set and analyzing it. [7].

Another category of data anomalies is the one that presents a specific and repetitive pattern over time, including fluctuations in their values. Any deviation from this pattern can be considered an anomaly [8].

Finally, some data behaviors are considered anomalies under conditions. A typical example is a bottleneck in an industrial network regarded as normal behavior during industrial working hours, such as in the morning or noon, but late at night is not normal and is an anomaly for network traffic flow. So, in this type of anomaly, the data values and the conditions that characterize them are essential [9, 10].

The industrial systems that are usually involved in the production process of a unit show a gradual deviation from the regular operation and not instantaneous failure. This makes it possible to predict deviant behavior, as there is a time interval between faults. As it is easily understood, the development of methods to detect anomalies is significant. They reduce the chances of an unexpected failure of the industrial system, which can have huge costs. [11].

All the abovementioned reasons led to the orientation of many research works on methods based on data analysis to detect abnormalities in the operation of industrial equipment. Based on the literature, detecting anomalies in a function can be done with statistical methods, but machine learning algorithms are also of particular interest.

## 2. Literature Review

The research community is continuously trying to implement machine learning technologies to take advantage of its unique characteristics related to anomaly detection, especially in environments that tend to produce extremely high amounts of data, like IIoT [1]. This section presents some recent studies in this field, some of which propose the relatively new Federated Learning framework.

Shah et al. [3] in 2018 investigated various machine learning algorithms for detecting anomalies in IIoT data from motor equipment. They analyzed the sensor data on fuel consumption, engine load, and oil pressure to determine when a certain engine exhibits anomalous behavior and may fail. To discover aberrations in machine behavior, they used multivariate linear regression, Gaussian mixture models, and time-series data analysis. To conclude their research, they employed simple statistical analysis to answer some of these scenarios, while machine learning algorithms were applied in others.

The article "Online Anomaly Detection of Industrial IoT Based on Hybrid Machine Learning Architecture" was retracted in 2023. Reasons: signs of a paper mill; suspected computer-generated content; unreliable results or conclusions; concerns about the data.

Zhou et al. [4] offered an overview of existing network anomaly detection algorithms as well as a brief description of the requirements and obstacles in IIoT network security. They also presented alternative anomaly detection approaches specifically suitable to IIoT networks. Such methods take advantage of the physical world's deterministic properties to find anomalies in observed behavior. The approaches based on specification descriptions and physical process modeling consider the operating dynamics of the underlying physical system and discover abnormalities from essential system characteristics. These techniques can be used in conjunction with cyber security techniques that detect anomalies caused by data modification. Finally, they proposed that for IIoT network anomaly detection, integrated cyber security and physical state estimate techniques would be more successful.

Four popular SCADA IIoT protocols, as well as their security flaws, were described by Zolanvari et al. [12]. Following that, they conducted a risk audit of the most significant and common security issues in IIoT systems and how machine learning-based solutions could assist in mitigating them. They showed a use case that included a real-world testbed constructed to perform cyber-attacks and designed an intrusion detection system. They used real-world cyber-attacks against this system to demonstrate how machine learning could address the identified gap by effectively handling them and measured the performance using representative measures to provide a fair assessment of the methods' effectiveness. Finally, feature priority ranking was investigated to emphasize the most important characteristics in separating malicious from normal traffic.

To fight against malicious actors, Yan et al. [13] presented a Hinge classification algorithm based on mini-batch gradient descent with an adaptive learning rate and momentum (HCA-MBGDALRM) in 2020. They stated that their method outperformed established approaches in terms of scalability and speed for deep network training. They also fixed the data skew issue during the shuffle phase. They developed a parallel framework for HCA-MBGDALRM to speed up the analysis of large traffic data volumes and enable IIoT safety improvements. Finally, they found that their technique increased the model's training efficiency and accuracy, ensuring the reliability of big data networking in IIoT.

The article "Online Anomaly Detection of Industrial IoT Based on Hybrid Machine Learning Architecture" was retracted in 2023. Reasons: signs of a paper mill; suspected computer-generated content; unreliable results or conclusions; concerns about the data.

Liu et al. [14] proposed the federated learning (FL) framework, which allows for decentralized edge devices to collaborate to train a deep anomaly detection (DAD) model, improving its generalization capabilities. They also developed a convolutional neural network long short-term memory (CNN- LSTM) model for detecting anomalies. They used their units to capture fine-grained characteristics, while maintaining the LSTM unit's benefits in forecasting time series data. The findings confirmed that their approach could maintain appropriate precision across all data sets and that the technique could enhance information flow 300 times without making any mistakes by reducing gradients. They even proposed a gradient compression mechanism to lower communication expenses and increase communication efficiency in order to accomplish real-time and lightweight anomaly detection.

Finally, Wang et al. [15] in 2021 suggested an anomaly detection system for IIoT, which utilized federated learning to improve confidentiality for various IIoT applications. They used this method to create a universal anomaly detection concept, training each local model using the deep reinforcement learning technique without aggregating local data sets to protect confidentiality. Their solution had the advantage of not requiring local data sets during federated learning, which decreased the risk of privacy compromise. The federated deep reinforcement learning algorithm then adequately identified anomalous users. The proposed technique demonstrated positive outcomes in diverse IIoT scenarios, according to the validation studies.

The proposed approach of this work aims at detecting signs of equipment behavior change in real-time to identify anomalies before the collapse of a system, which may be due to damage or cyber-attacks [16].

## 3. Proposed Methodology

The primary idea of the proposed methodology is based on the logic of the P–F curve, which gives a representative picture of the behavior of equipment in regular operation and in that which presents abnormalities [8]. Therefore, the aim is to predict the point at which the behavior of the equipment begins to change (point P) much earlier than would be perceived by the person in charge of the operation of the equipment from indications that would appear. The technological innovations related to sensors contribute to achieving the abovementioned goal for monitoring the production process and then recording the data necessary for the subsequent analysis by the proposed hybrid machine learning system [7].

The article "Online Anomaly Detection of Industrial IoT Based on Hybrid Machine Learning Architecture" was retracted in 2023. Reasons: signs of a paper mill; suspected computer-generated content; unreliable results or conclusions; concerns about the data.

More specifically, the proposed approach contains three basic algorithms. The first implements a long short-term memory (LSTM) neural network [17], the next implements the time-domain feature extraction process, and the last is the Bayesian online changepoint detection [18]. Initially, the measurements recorded in real-time by the sensors are taken as input from the LSTM neural network, and the predicted values for the exact quantities are generated in a period predetermined by the network composition. These values then feed the algorithm to extract the features needed for the upcoming data analysis. It is also important to note that the data taken as input to this process are not the sum of the data of each size but are selected from a time-varying fixed-size window [19]. Finally, the signal resulting from the output of the power supplies the change point detection algorithm, which indicates through a graph the probability that a point is a change point. At the same time, through the probabilities that it calculates, it predicts the future state of the equipment in the period above determined by the neural network. This procedure is followed because the change point detection algorithm is sensitive to noise and should be subtracted from the signal to be inserted into it to output information at a higher level than the original data and reduce the uncertainty it initially includes [20].

### 3.1. Long Short-Term Memory Neural Network

LSTM neural networks can retrieve information from a significant number of past time steps, providing satisfactory results in problems with serial data and especially time series. It is a chain of similar neural devices, but each consists of four interact levels. The synthesis and function of the basic structures of an LSTM cell can be attributed to steps as follows [17, 21, 22]:

The output of the last cell and the current input to the cell are combined in one vector, where it concerns all the data to be processed:

(1) $$\begin{array}{c} \left[h_{t-1}+x_{t}\right]. \end{array}$$

The above vector goes through the “forget gate,” and the following function is generated:

(2) $$\begin{array}{c} f_{t}=\sigma \left(W_{f}*\left[h_{t-1},x_{t}\right]+b_{f}\right). \end{array}$$

This function is multiplied by the previous memory state so that we obtain the following:

(3) $$\begin{array}{c} \left[C_{t-1}*f_{t}\right]. \end{array}$$

The vector [*h*_*t*−1_+*x*_*t*_] passes through the “input gate,” and the following function is generated:

(4) $$\begin{array}{c} i_{t}=\sigma \left(W_{i}*\left[h_{t-1},x_{t}\right]+b_{i}\right). \end{array}$$

The same vector passes through the tanh function and produces the following:

(5) $$\begin{array}{c} {\tilde{C}}_{t}=\text{tanh}\left(W_{C}*\left[h_{t-1},x_{t}\right]+b_{C}\right). \end{array}$$

The results of the previous two steps are multiplied by each other to obtain the following:

(6) $$\begin{array}{c} \left[\begin{array}{c} i_{t}*{\tilde{C}}_{t} \end{array}\right]. \end{array}$$

Adding the results produced by the multiplications in the above steps results in a new memory state:

(7) $$\begin{array}{c} C_{t}=C_{t-1}*f_{t}+i_{t}*{\tilde{C}}_{t}. \end{array}$$

The vector [*h*_*t*−1_+*x*_*t*_] passes through the “output gate,” and the following function is generated:

(8) $$\begin{array}{c} o_{t}=\sigma \left(W_{o}*\left[h_{t-1},x_{t}\right]+b_{o}\right). \end{array}$$

The new memory state operates as a tanh function, and the result is multiplied by the above function producing the new cell output:

(9) $$\begin{array}{c} h_{t}=o_{t}*\text{tanh}\left(C_{t}\right). \end{array}$$

The article "Online Anomaly Detection of Industrial IoT Based on Hybrid Machine Learning Architecture" was retracted in 2023. Reasons: signs of a paper mill; suspected computer-generated content; unreliable results or conclusions; concerns about the data.

### 3.2. Feature Extraction

The data collected by sensors usually require a pre-treatment to remove the noise contained in the signal due to their use and minimize the uncertainty caused by them. In addition, in this way, information is produced with sufficient accuracy so that the analysis of the data subsequently produces reliable results. Especially in vibration signals, such as those made mainly in industry, the extraction of characteristic quantities is necessary when the data analysis involves the detection of errors and the prediction of various quantities [23].

The method used to extract feature sizes is done in the time-domain features extraction. These characteristics refer to the mean, which calculates the quotient resulting from the sum of the signal values and their number. The root mean square (RMS) calculates the square root of the mean value of the signal raised to the square. This size increases gradually as an error develops within the signal to be studied, but it cannot provide information at the initial stage of error development [20, 24, 25]. In addition, variance is a quantity that indicates the scatter of the signal using the mean as a reference. In contrast, standard deviation (std) determines the square root of the signal variance. More specific sizes, capable of delivering more information, are kurtosis and skewness, which process the probability density function of the signal. More specifically, kurtosis calculates the maximum value of the function and indicates whether the signal can respond immediately to a change. Under normal conditions, the kurtosis emitted by a vibration signal is approximately equal to a pre-agreed value, e g., three. At the same time, if there are errors in it, then the probability density function changes, and therefore, the value of the curvature is greater than that of regular operation. Accordingly, skewness is a quantity obtained from the mean value of the probability density function and is used to indicate whether the vibration signal is negatively or positively skewed. In a signal with normal distribution, the skewness has zero value. Still, if it is disturbed due to errors, then it will receive either a negative or a positive value depending on the skewness it will present. In addition, it is worth noting that the abovementioned two values can be applied to signals that are not purely continuous in time (stationary) in contrast to characteristics such as mean and standard deviation [26, 27].

The article "Online Anomaly Detection of Industrial IoT Based on Hybrid Machine Learning Architecture" was retracted in 2023. Reasons: signs of a paper mill; suspected computer-generated content; unreliable results or conclusions; concerns about the data.

Another quantity that can be deduced from the probability density function for vibration signals is entropy, which calculates the histogram of the above function and indicates the magnitude of the randomness and uncertainty of the signal. Finally, the lower and upper bound histograms belong to the same category, which calculates the maximum and minimum values of the probability density function, respectively [18, 28].

The abovementioned are the appropriate characteristics for processing vibration signals coming from the industrial sector. Also, the attributes in question result in a value calculated from the total of the data studied. However, in this approach, the feature extraction process is rolling, and the result obtained is a curve with the values calculated at each step. In other words, this process uses a window of a specific size so that the calculation of features is not done from the whole data set but from a subset of a fixed size that moves over time. Therefore, the analysis of the exported characteristics includes values from previous times and the current one. The amount of these historical data is determined by the window set for calculating each attribute. The use of the window and therefore, the historical data result in the extraction of information at a higher level and greater computational efficiency [7, 24, 29].

The work used sliding windows, and the exact window size for each feature was determined after testing to achieve the best result in terms of information to be extracted from the feature display.

### 3.3. Bayesian Online Changepoint Detection

A time series is a collection of observations in chronological order. These data are large, so they take up more memory, are multidimensional, and are constantly updated. Another characteristic of them is abrupt changes in their structure, such as a jump in a much higher value than the previous one or a different behavior in data distribution. Those points that change behavior is called change points and essentially split the data into homogeneous parts. Detection abnormalities in a state of operation is a process in which abrupt changes in serial data are identified and performed in real-time or afterward. Most algorithms with “Bayesian” logic focus on the fragmentation of the data set and on techniques that produce results from their subsequent analysis. Still, the algorithm used in this study focuses on identifying the cause of the problem. During execution, it creates a distribution of the next value in the data sequence, taking into account only the values that have been recorded so far. This approach is suitable for detecting points of change in time series due to its ease in quantifying the probability that a position is a point of difference [10, 21, 30].

The article "Online Anomaly Detection of Industrial IoT Based on Hybrid Machine Learning Architecture" was retracted in 2023. Reasons: signs of a paper mill; suspected computer-generated content; unreliable results or conclusions; concerns about the data.

The quantities to be studied are a series of time-determined observations divided into various dissimilar and non-overlapping areas with a specific length. At the same time, the boundaries between them are the changepoints. It is also considered that these observations are independent and uniformly distributed random variables with probability distribution *P*(*x*_*t*_*|n*_*ρ*_) where *n*_*ρ*_ are independent and similarly distributed random variables. In addition, a grouping of observations between time instant *a* and *b* is denoted by *x*_a b_ and the preset probability distribution in the space between two change points with *P*_gap_(*g*).

This approach estimates the subsequent probability distribution at the current data length *r*_*t*_ at time *t*. Data length *r*_*t*_ is a time-dependent function, which is zeroed when a state change occurs, i e., it encounters a change point and refers to the data set from the most recent change point to that time point. In addition, the observations concerning a data length *r*_*t*_ are denoted by (*r*), while if the data length is zero (*r*  = 0), then they are denoted by *x*^(*r*)^ .

To predict the probability distribution at the current data length, the ex-post probability distribution must first be calculated retrospectively, and the marginal prediction distribution through the following formulas must be integrated into it [24, 31, 32]:

(10) $$\begin{array}{c} P\left(x_{t+1}|x_{1:t}\right)=\sum_{r_{t}}P\left(x_{t+1}|x_{t}^{\left(r\right)},r_{t}\right)P\left(r_{t}|x_{1:t}\right)\\ P\left(r_{t}|x_{1:t}\right)=\frac{P\left(r_{t},x_{1:t}\right)}{P\left(x_{1:t}\right)}\\ P\left(r_{t},x_{1:t}\right)=\sum_{r_{t-1}}P\left(r_{t},r_{t-1},x_{1:t}\right). \end{array}$$

The formula *P*(*r*_*t*_, *x*_1:*t*_) calculates the probability density function in the current data length retrospectively to calculate the ex-post probability distribution. Finally, it is worth noting that the forecast distribution depends only on recent data (*r*). Therefore, the probability density function can be calculated retrospectively based on the current data length *r*_*t*_, given *r*_*t*__−1_, and the predictive distribution results from the new value observed, given the values observed so far.

The article "Online Anomaly Detection of Industrial IoT Based on Hybrid Machine Learning Architecture" was retracted in 2023. Reasons: signs of a paper mill; suspected computer-generated content; unreliable results or conclusions; concerns about the data.

To calculate the abovementioned quantities and formulate retrospective formulas, it is necessary to define the limit conditions based on two considerations. In the first case, a point change has occurred before the first value of the data to be studied, and therefore, the probability function is zeroed for the initial data length. In the second case, on the other hand, the study is done on a recent subset of data, and the boundary condition is formed by the normalized survival function, which indicates the time at the end of which one or more events occur. The conditions in the mathematical form are shown below [25, 33, 34]:

(11) $$\begin{array}{c} P\left(r_{0}=0\right)=1\\ P\left(r_{0}=\tau \right)=\frac{1}{Z}\tilde{S}\left(\tau \right), \end{array}$$

where *Z* is the normalized constant and $\tilde{S}\left(\tau \right)=\sum_{t=r+1}^{\infty }P_{\text{gap}}\left(g=t\right).$

The computational efficiency of the algorithm is due to the form of the probability function that there is a point of change based on previous data. This function is zero everywhere except when the data length increases as a new value are added to it and when a unique change point is observed. The function of this probability is shown below [18], [35]:

(12) $$\begin{array}{c} P\left(r_{t}|r_{t-1}\right)=\left\{\begin{array}{c} H\left(r_{t-1}+1\right),r_{t}=0\\ 1-H\left(r_{t-1}+1\right),r_{t}=r_{t-1}+1\\ 0,\text{elsewere} \end{array},\right. \end{array}$$

where H(t) is the hazard function and represents which pieces of data have a higher or lower probability of an event occurring and is equal to

(13) $$\begin{array}{c} H\left(\tau \right)=\frac{P_{gap}\left(g=\tau \right)}{\sum_{t=\tau }^{\infty }P_{gap}\left(g=t\right)}. \end{array}$$

The exponential models are a handy tool for detecting anomalies and essentially for the algorithm described in this work. They are easy to use because they can offer a set of parametric probability distributions and statistical quantities, which can be calculated during data collection. The probability format based on these models is reported for completeness and is shown in the following equations [36], [37]:

(14) $$\begin{array}{c} H\left(\tau \right)=\frac{P_{gap}\left(g=\tau \right)}{\sum_{t=\tau }^{\infty }P_{gap}\left(g=t\right)}\\ P\left(x|n\right)=h\left(x\right)\text{exp}\left(n^{T}U\left(x\right)-A\left(n\right)\right.\\ A\left(n\right)=\text{log}\int \text{d}nh\left(x\right)\text{exp}\left(n^{T}U\left(x\right)\right) \end{array}$$

The article "Online Anomaly Detection of Industrial IoT Based on Hybrid Machine Learning Architecture" was retracted in 2023. Reasons: signs of a paper mill; suspected computer-generated content; unreliable results or conclusions; concerns about the data.

## 4. Data Set, Scenarios, and Results

Data from an industrial plant that performs cold rolling on metals were used for the present study. This process substantially reduces the thickness of the metal to the optimum smaller thickness with a perfectly smooth surface or reshapes it through two rollers, which rotate in the opposite direction from that of the metal. The metal temperature must be lower than where the metal recrystallizes to do this process.

Ten sensors have been installed in the cold rolling equipment to collect data on vibrations to implement the experiments. Also, in the cold rolling unit, there is a sensor that measures the speed of the motor and another that measures its current. In this study, we are only interested in the data collected by the former. In more detail, these sensors record values for four different variables every ten seconds for vibration data. These are the acceleration, the state of the rollers in terms of resistance and vibration (overall bearing), the abrupt change of state (shock), and the speed (velocity). These measurements cover ten months, and the number of files created by different sensors was ten in number, with a size ranging from 870,000 to 990,000 particles of data.

Each of the re-created files contains six columns, the first of which refers to the name of the roller, depending on the position of the sensor in it. The second column has the date and time in timestamp UTC so that it is expressed globally and not locally, and the other four columns refer to the values of the quantities produced by the sensors, and these data are time series. From the statistical analysis of the data, it initially appears that the magnitude “shock” describes the existence or not of a significant disturbance in the operation of the device. Its non-existence is illustrated with a zero value while the opposite state with a positive value. The acceleration takes only positive values with a minimum value close to zero while the maximum does not exceed 7. Similar behavior is shown by the second size overall bearing, with its maximum value not exceeding 8. Finally, velocity indicates that the minimum price is close to 0, but its maximum value is much higher than the two previous sizes. An indicative representation of the sizes in question is presented in Figure 1.

The diagrams above show the data for each of the quantities recorded by the sensor. From the figure regarding acceleration, we observe a value that differs from the rest but allows us to see the variation of the other values, as there is no considerable difference between the maximum and the rest. If we capture some values before this maximum value, as shown in the velocity figure on the right, we will notice a difference between the speed data, and they are not zero. In the case of velocity, on the other hand, it is evident that the fluctuation of the values does not exist, and they are all presented as a straight line very close to zero, which is interrupted by a vertical that represents the maximum value. The high-velocity value probably comes from a disturbance in the sensor environment. It is not interpreted in a natural way to be related to the behavior of the equipment [9, 29, 33].

The article "Online Anomaly Detection of Industrial IoT Based on Hybrid Machine Learning Architecture" was retracted in 2023. Reasons: signs of a paper mill; suspected computer-generated content; unreliable results or conclusions; concerns about the data.

The experimental process aims to detect anomalies in the industrial data. The diagrammatic representation of the experiment is shown in Figure 2.

Acceleration, overall bearing, and velocity values are predicted via the LSTM neural network during the experimental process. In the intermediate stage of the process, the characteristics are extracted from vibration signals (raw data) in the time domain. The procedure concerns the following sizes [17, 20, 21, 27]:

(15) $$\begin{array}{c} \text{mean}=\frac{\sum_{i=1}^{N}x_{i}}{N}\\ \text{RMS}=\sqrt{\frac{1}{N}\sum_{i=1}^{N}x_{i}^{2}}\\ \text{STD}=\sqrt{\frac{\sum_{i=1}^{N}{\left(x_{i}-m\right)}^{2}}{\left(N-1\right)\sigma^{2}}}\\ \text{var}=\frac{\sum_{i=1}^{N}{\left(x_{i}-m\right)}^{2}}{\left(N-1\right)\sigma^{2}}\\ Ku=\frac{\sum_{i=1}^{N}{\left(x_{i}-m\right)}^{4}}{\left(N-1\right)\sigma^{4}}\\ Sk=\frac{\sum_{i=1}^{N}{\left(x_{i}-m\right)}^{3}}{\left(N-1\right)\sigma^{3}}\\ e\left(p\right)=-\sum_{i=-1}^{n}p\left(z_{i}\right){\text{log}}_{2}p\left(z_{i}\right)\\ h_{U}=\text{max}\left(x_{i}\right)+\frac{\Delta }{2}\\ h_{L}=\text{max}\left(x_{i}\right)-\frac{\Delta }{2}, \end{array}$$

which are used to detect differences between vibration signals.

Then, the feature extraction algorithm is applied, producing five rolling features. Specifically, let *τ*_*0*_∈*T* be the time of submission of the relevant duration query, then the scope of a rolling window with width *ω* and step *δ* for each *τ*∈ *T* (with *τ* ≥ *t*0) extends [19, 30]:

(16) $$\begin{array}{c} {\text{scopes}}_{s}\left(\tau ,\omega ,\delta \right)=\left\{\begin{array}{c} \left[\tau -\omega +1,\tau \right],\alpha v\tau \geq \tau_{0}+\omega \wedge \text{mod}\left(\left(\tau -\tau_{0}\right),\delta \right)=0\\ {\text{scope}}_{s}\left(\tau -1,\omega ,\delta \right),\alpha v\text{mod}\left(\left(\tau -\tau_{0}\right),\delta \right)\neq 0\\ \left[\tau_{0},\tau \right],\alpha v\tau_{0}\leq \tau <\tau_{0}+\omega \wedge \text{mod}\left(\left(\tau -\tau_{0}\right),\delta \right)=0 \end{array},\right. \end{array}$$

where the magnitudes *τ*_*0*_, *τ*∈*T* are expressed in time landmarks and *ω*, *δ*∈*ℕ* are expressed in a range of time intervals (*ω, δ* > 0). For the sake of simplicity, the abovementioned definition implies that all-time quantities are expressed as natural numbers so that the function is calculated at distinct time points of *T*. Then, the window multiples result from the relation [19, 38]:

(17) $$\begin{array}{c} W_{s}\left(S,\tau ,\omega ,\delta \right)=\left\{s\in S\left(\tau \right):s.A_{\tau }\in {\text{scope}}_{s}\left(\tau ,\omega ,\delta \right)\right\}. \end{array}$$

Usually, step *δ* is the same size as the unit of time (e g., second) so that the window's progress is ideally in line with the corresponding time. Because *δ*<*?* is generally valid, the contents of two consecutive snapshots of the popup window overlap. Meanwhile, its contents remain unchanged until the function is applied again to the next pulse, after *δ* time. This is expressed by the retroactive expression in the middle branch of the function: the edges of the window change only at times specified in step *δ*. The third part of the function provides the possibility of initial “missing” windows immediately after the query when the range exceeds the time range of the current contents.

The article "Online Anomaly Detection of Industrial IoT Based on Hybrid Machine Learning Architecture" was retracted in 2023. Reasons: signs of a paper mill; suspected computer-generated content; unreliable results or conclusions; concerns about the data.

Since the range function is monotonous due to the evolution of time implies a homologous passing of the intervals and can be defined even for future moments. All the following elements of the current are covered, regardless of when and if they finally appear. For example, suppose the kurtosis attribute is exported with window = 25. In that case, the first value of this attribute will be extracted from the data to be studied in positions 1 to 25, while the second value from the data in positions 2 to 26 and so on. The term position means the order in which the data from the sensor have been recorded in this case.

Finally, for each time *τ*∈*T*, the window connection operator returns the joining of pairs of blocks that appear in the respective window snapshots [19]:

(18) $$\begin{array}{c} S_{1}\left(\tau \right)\infty S_{2}\left(\tau \right)=\left\{\left(s_{1},s_{2},\tau_{m},:s_{1}\in W_{1}\left(S_{1}\left(\tau \right)\right),s_{2}\in W_{2}\left(S_{2}\left(\tau \right)\right)\wedge \right.\right.\\ \left.\wedge E\left(s_{7},s_{2}\right)\wedge \tau_{m}=max\left(s_{1},A_{\tau },s_{2},A_{\tau }\right)\right\}. \end{array}$$

It is essentially a sliding-window join process, separately for each stream. Each new input block of current *S*_*1*_ is checked for connection condition *E* with all existing rolling window *W*_*2*_ of the stream *S*_*2*_. The exported results receive the most recent timeline displayed in the primary tuples pair if matching elements are found. This is, after all, the time indicated that restores the order of the final results of the generated data stream.

The article "Online Anomaly Detection of Industrial IoT Based on Hybrid Machine Learning Architecture" was retracted in 2023. Reasons: signs of a paper mill; suspected computer-generated content; unreliable results or conclusions; concerns about the data.

The Bayesian online changepoint detection algorithm [20] is then applied to each of the characteristics generated for each size studied to detect a change in equipment operation through feature analysis. This process can be captured in the following steps [17, 20, 39]:

**Step 1 .**

Initialization through following marginal conditions:

(19) $$\begin{array}{c} P\left(r_{0}\right)=\tilde{S}\left(r\right)\text{or}P\left(r_{0}=0\right)=1\\ v_{1}^{\left(0\right)}=v_{\text{prior}}\\ X_{1}^{\left(0\right)}=X_{\text{prior}}. \end{array}$$

**Step 2 .**

Observation of the following data value.

**Step 3 .**

Predictive probability estimation as follows:

(20) $$\begin{array}{c} \pi_{t}^{\left(r\right)}=P\left(x_{t}|v_{t}^{\left(r\right)},X_{t}^{\left(r\right)}\right). \end{array}$$

**Step 4 .**

Probability calculation as the current data length increases as shown below:

(21) $$\begin{array}{c} P\left(r_{t}=r_{t-1}+1,x_{1:t}\right)=P\left(r_{t-1},x_{1:t-1}\right)\pi_{t}^{\left(r\right)}\left(1-H\left(r_{t-1}\right)\right). \end{array}$$

**Step 5 .**

Calculation of probability for the existence of a point of change as follows:

(22) $$\begin{array}{c} P\left(r_{t}=0,x_{1:t}\right)=\sum_{r_{t-1}}P\left(r_{t-1},x_{1:t-1}\right)\pi_{t}^{\left(r\right)}H\left(r_{t-1}\right). \end{array}$$

**Step 6 .**

Probability calculation in the observation group, from the first to the time *t*:

(23) $$\begin{array}{c} P\left(x_{1:t}\right)=\sum_{r_{t}}P\left(r_{t},x_{1:t}\right). \end{array}$$

**Step 7 .**

The data length distribution is defined as follows:

(24) $$\begin{array}{c} P\left(r_{t}|x_{1:t}\right)=\frac{P\left(r_{t},x_{1:t}\right)}{P\left(x_{1:t}\right)}. \end{array}$$

**Step 8 .**

The parameter value as shown below:

(25) $$\begin{array}{c} v_{t+1}^{\left(0\right)}=v_{\text{prior}}\\ X_{t+1}^{\left(0\right)}=X_{\text{prior}}\\ v_{t+1}^{\left(r+1\right)}=v_{t}^{\left(r\right)}+1\\ X_{t+1}^{\left(r+1\right)}=X_{t}^{\left(r\right)}+u\left(x_{t}\right). \end{array}$$

**Step 9 .**

Calculation of the marginal forecast distribution:

(26) $$\begin{array}{c} P\left(x_{t+1}|x_{1:t}\right)=\sum_{r_{t}}P\left(x_{t+1}|x_{t}^{\left(r\right)},r_{t}\right)P\left(r_{t}|x_{1:t}\right). \end{array}$$

**Step 10 .**

Return to observe the next value.

The temporal and spatial complexity of the algorithm is linear about the amount of data to be processed and is calculated at each time point based on the data observed so far. The abovementioned description gives a clear picture of the operation and purpose of the algorithm, which calculates the quantities required to calculate the probability that each point is a change point (log-likelihood). In particular, the algorithm accepts as input the data in which it is desirable to detect anomalies and, as a result, is initially extracted for each time corresponding to the data set, the value of the probability to be a point of change. These values are used to create the diagram that presents the above information graphically. More specifically, the values of the probabilities that are calculated refer to the size log-likelihood, which has a logarithmic character and a negative sign. The vertical axis is on a logarithmic scale in the diagram formed, and the horizontal one represents time.

The article "Online Anomaly Detection of Industrial IoT Based on Hybrid Machine Learning Architecture" was retracted in 2023. Reasons: signs of a paper mill; suspected computer-generated content; unreliable results or conclusions; concerns about the data.

Another quantity that results from applying the algorithm is the position of the point most likely to be a point of change. Although the generated curve may have enough points with a sufficient probability value to show a state change, the algorithm returns the highest probability value, i e., the point where the curve is at the highest position on the chart. This approach returns to the time when behavior change is most likely. Finally, it returns the average values found in all previous time points from the algorithm's most probable for a state change. Similarly, the average size values studied and found after the aforementioned time are calculated.

The results of the above experiment are shown in the following diagrams. The first row of the figures shows the predicted values of the interest quantities compared to the actual values of these data. The mode of each feature is different, having the same input. Of course, there are several similarities in the attributes mean, std and rms. Therefore, the result of the algorithm shows several common points for the specific features. In addition to all the diagrams showing the result of the experiment, a clear picture of the process of detecting anomalies is demonstrated as the peaks of the curves are clear.

Below are the results for some data sets where the procedure of this experiment was applied. In each figure, the first column presents the initial data of each size from acceleration, overall bearing, and velocity for a data set. The following columns show the algorithm's result for each kurtosis feature, skewness, mean, std, and rms. These curves are the result to be evaluated in the experiment. The results show the recording of the time where the point of change of the equipment operates according to the algorithm is considered. The value forecast was made with a time limit of half an hour.

The article "Online Anomaly Detection of Industrial IoT Based on Hybrid Machine Learning Architecture" was retracted in 2023. Reasons: signs of a paper mill; suspected computer-generated content; unreliable results or conclusions; concerns about the data.

Finally, an important observation is that applying the algorithm to the characteristics mean, standard deviation, and rms gives better results about kurtosis and skewness. While they exhibit similar behavior, they are different for each data set, and this can be perceived from the time they identify as the most likely to occur abnormalities. In addition, the mean feature realizes earlier the malfunction of the equipment as it presents an anomaly at a previous time from the other elements for all the sizes studied.

## 5. Conclusions

The detection and timely assessment of abnormalities in the operation of the industrial ecosystem allows the detection of incidents and the corresponding identification of correlations and causal relationships with security incidents, which can significantly mitigate the effects of sophisticated cyber-attacks. In this spirit, a hybrid system of deep machine learning architecture was used to predict anomalies in the operation of industrial equipment. Specifically, the Bayesian online changepoint detection algorithm was used to detect anomalies, the time-domain features extraction process for feature extraction, and the long-short term memory neural network to predict the values of the magnitudes that reflect the correct or not the operation of the equipment. Sensors in real-time record the data used. Because they contain a lot of noise, detecting anomalies without prior pre-treatment produces excellent uncertainty. If the detection is done after the proper pre-processing of the data, the results are distinguished with great accuracy.

Future developments of the work concern the development of more complex deep learning architectures to model the problem more fully in question. Procedures should also be studied to add other parameters as input and improve the model's accuracy and efficiency. At the same time, predictive analysis procedures for new methods that will fully automate extracting data characteristics and detecting anomalies should be studied.

## Figures and Tables

**Figure 1:** Depiction of the data set (random state).

**Figure 2:** Flowchart of the proposed anomaly detection process.

## Data Availability

The data used to support the findings of this study are available from the corresponding author upon reasonable request.

## References

[1] Banafa A. (2018). 2 the industrial Internet of Things (IIoT): challenges, requirements and benefits. *Secure and Smart Internet of Things (IoT): Using Blockchain and AI*.

[2] Schneider S. (2017). THE INDUSTRIAL INTERNET OF THINGS (IIoT). *Internet of Things and Data Analytics Handbook*.

The article "Online Anomaly Detection of Industrial IoT Based on Hybrid Machine Learning Architecture" was retracted in 2023. Reasons: signs of a paper mill; suspected computer-generated content; unreliable results or conclusions; concerns about the data.

[3] Shah G., Tiwari A. Anomaly detection in IIoT.

[4] Zhou L., Guo H. Anomaly detection methods for IIoT networks.

[5] Mumtaz S., Alsohaily A., Pang Z., Rayes A., Tsang K. F., Rodriguez J. (2017). Massive Internet of Things for industrial applications: addressing wireless IIoT connectivity challenges and ecosystem fragmentation. *IEEE Industrial Electronics Magazine*.

[6] Sulaiman S., Aldeehani A., Alhajji M., Aziz F. A. (2021). Development of integrated supply chain system in manufacturing industry. *Journal of Computational Methods in Science and Engineering*.

[7] Chalapathy R., Chawla S. (2019). Deep learning for anomaly detection: a survey. http://arxiv.org/abs/1901.03407.

[8] Al Jallad K., Aljnidi M., Desouki M. S. (2020). Anomaly detection optimization using big data and deep learning to reduce false-positive. *Journal of Big Data*.

[9] Cuzzocrea A. Big data lakes: models, frameworks, and techniques.

[10] Xing L., Demertzis K., Yang J. (2020). Identifying data streams anomalies by evolving spiking restricted Boltzmann machines. *Neural Computing & Applications*.

[11] Boubekeur M. Industrial applications for cyber-physical systems.

[12] Zolanvari M., Teixeira M. A., Gupta L., Khan K. M., Jain R. (2019). Machine learning-based network vulnerability analysis of industrial Internet of Things. *IEEE Internet of Things Journal*.

[13] Yan X., Xu Y., Xing X., Cui B., Guo Z., Guo T. (2020). Trustworthy network anomaly detection based on an adaptive learning rate and Momentum in IIoT. *IEEE Transactions on Industrial Informatics*.

[14] Liu Y., Kumar N., Xiong Z., Lim W. Y. B., Kang J., Niyato D. Communication-efficient federated learning for anomaly detection in industrial Internet of Things.

[15] Wang X., Garg S., Lin H. (2021). Towards accurate anomaly detection in industrial internet-of-things using hierarchical federated learning. *IEEE Internet of Things Journal*.

[16] Tsiknas K., Taketzis D., Demertzis K., Skianis C. (2021). Cyber threats to industrial IoT: a survey on attacks and countermeasures. *IoT*.

[17] Wu D., Jiang Z., Xie X., Wei X., Yu W., Li R. (2020). LSTM learning with bayesian and Gaussian processing for anomaly detection in industrial IoT. *IEEE Transactions on Industrial Informatics*.

[18] del Águila I. M., del Sagrado J. (2016). Bayesian networks for enhancement of requirements engineering: a literature review. *Requirements Engineering*.

[19] Baig S. u. R., Iqbal W., Berral J. L., Carrera D. (2020). Adaptive sliding windows for improved estimation of data center resource utilization. *Future Generation Computer Systems*.

[20] van de Schoot R., Depaoli S., King R. (2021). Bayesian statistics and modelling. *Nature Reviews Methods Primers*.

The article "Online Anomaly Detection of Industrial IoT Based on Hybrid Machine Learning Architecture" was retracted in 2023. Reasons: signs of a paper mill; suspected computer-generated content; unreliable results or conclusions; concerns about the data.

[21] Guo Y. Stock price prediction based on LSTM neural network: the effectiveness of news sentiment analysis.

[22] Orozco C. I., Buemi M. E., Berlles J. J. Towards an attention mechanism LSTM framework for human action recognition in videos.

[23] Chitty-Venkata K. T., Somani A. Impact of structural faults on neural network performance.

[24] Anderson T. W. (2003). *An Introduction to Multivariate Statistical Analysis*.

[25] Bevington P., Robinson D. K. (2003). *Data Reduction and Error Analysis for the Physical Sciences*.

[26] Conradi C., Pantea C., Robeva R., Macauley M. (2019). Multistationarity in biochemical networks: results, analysis, and examples. *Algebraic and Combinatorial Computational Biology*.

[27] Raschka S. (2014). An overview of general performance metrics of binary classifier systems. http://arxiv.org/abs/1410.5330.

[28] Ahmadlou M., Adeli H. (2010). Enhanced probabilistic neural network with local decision circles: a robust classifier. *Integrated Computer-Aided Engineering*.

[29] D’Acquisto G., Domingo-Ferrer J., Kikiras P., Torra V., de Montjoye Y.-A., Bourka A. (2015). Privacy by design in big data: an overview of privacy enhancing technologies in the era of big data analytics. https://arxiv.org/abs/1512.06000.

[30] Tellis V. M., D’Souza D. J. Detecting anomalies in data stream using efficient techniques: a review.

[31] Hwang U., Park J., Jang H., Yoon S., Cho N. I. (2019). PuVAE: a variational autoencoder to purify adversarial examples. *IEEE Access*.

[32] Guopan S. The effect of probability on risk perception and risk preference in decision making.

[33] Alzubaidi L., Zhang J., Humaidi A. J. (2021). Review of deep learning: concepts, CNN architectures, challenges, applications, future directions. *Journal of Big Data*.

[34] Gupta S., Al-Obaidi S., Ferrara L. (2021). Meta-analysis and machine learning models to optimize the efficiency of self-healing capacity of cementitious material. *Materials*.

[35] Qian J., Lu J. P., Hui S. L., Ma Y. J., Li D. Y. (2015). Dynamic analysis and CFD numerical simulation on backpressure filling system. *Mathematical Problems in Engineering*.

[36] Berger J. O., Berger J. O. (1985). Bayesian analysis. *Statistical Decision Theory and Bayesian Analysis*.

[37] Derrick B., White P. (2017). Comparing two samples from an individual likert question. *International Journal of Mathematics and Statistics*.

[38] Amron M. T., Ibrahim R., Chuprat S. (2017). A review on cloud computing acceptance factors. *Procedia Computer Science*.

[39] Kingma D. P., Welling M. (2014). Auto-encoding variational bayes. http://arxiv.org/abs/1312.6114.

